The article "Construction of Online Teaching Acceptance Model of University Library under the Epidemic Situation" was published in 2022. Journal: J Environ Public Health.

# Construction of Online Teaching Acceptance Model of University Library under the Epidemic Situation

**DOI:** 10.1155/2022/5628711

**Published:** 2022-09-29

**Authors:** Nan Wu

**Affiliations:** Library, Heilongjiang University of Science and Technology, Harbin 150027, China

## Abstract

In order to improve the online teaching quality of university libraries, this paper puts forward the construction of the online teaching acceptance model of university libraries under the background of the epidemic situation, constructs the basic theoretical framework of the teaching evaluation system, establishes the basic evaluation indicators, takes the online teaching quality evaluation and the operability of the evaluation system as the constraint object, and determines the index parameter set after class review; the three modules were guided and trained. Based on the big data analysis of the evaluation index system, accurate teaching quality scores or grades were calculated, and the online teaching acceptance evaluation of university libraries was realized. The results of empirical analysis show that this method can realize the accurate evaluation of teaching quality, promote the deep integration of online teaching theory and practice in university libraries, and improve the acceptance level of online teaching quality.

## 1. Introduction

The sudden attack of novel coronavirus in 2019 has directly led to the delay of the spring opening of colleges and universities across the country in 2020. Students in colleges and universities across the country are isolated at home to fight against the virus [1, 2]. During the epidemic period, in order not to delay students' learning, the ministry of education advocated that all localities provide learning support for students through network technology, so as to “stop teaching and stop school”. In the process of school education, the online teaching course of university library always occupies an important position [3, 4]. It plays an important role in promoting students to form the core quality of library teaching, learn library skills, develop healthy behaviors, cultivate library ethics, and promote students' comprehensive development [5, 6]. During the epidemic period, online teaching courses of university libraries can improve students' physical and mental conditions and carry out online teaching education of university libraries, which is conducive to the safety of students through the isolation period and the comprehensive development of online teaching of university libraries [7, 8]. After the outbreak of the epidemic, the working mode of network teaching in university libraries has changed to some extent, from the previous offline service to the online service. In this case, the number of visits to the library's website has increased dramatically [9, 10]. Due to insufficient preparation, the network speed and the configuration of software and hardware facilities cannot keep up with each other, resulting in the jam of the electronic server, which seriously affects the access speed of teachers and students. With the increase of the number of visits, readers' demand for the types of electronic resources has also increased, and the original electronic resources can obviously not meet the needs of teachers and students.

Whether it is the basis of reality, the experience of online courses in China, or the future development of education, it is forced to speed up the construction of online teaching courses in university libraries. It can no longer be passively accepted that the construction of online courses in university libraries requires detailed planning, of which the teaching quality evaluation index system is the most important. Online teaching in university libraries is Internet distance education. It refers to educational activities that break through time and space constraints. It refers to activities that organize teaching and two-way interaction in classes. There are several common forms such as live teaching, video teaching, and live face-to-face teaching. It has been used as an auxiliary teaching method in the field of education. However, the outbreak of COVID-19 in 2020 ushered in a historic turning point for online teaching, which changed from the auxiliary teaching mode in the ordinary period to the main teaching mode in the epidemic period. As a temporary alternative to offline teaching, the education mode not only breaks the restrictions of time and space, saves teaching costs, and brings convenience to students' learning, but also attracts a large number of online education and learning users with its unique openness and flexibility, diversified online teaching modes of university libraries, rich teaching contents, and increasingly mature online teaching technologies. This not only shows that online education plays a positive role in the education of today's society, but also highlights its strong vitality and bright development prospects.

In addition, online teaching, as a product of the times, is the embodiment of the deep integration of modern information technology and education. Although it is not yet mature, it is a teaching method that cannot be ignored in the future. This research topic and research method not only ensure that this paper has strong theoretical support, but also make the research results have strong practical guiding significance. It provides reference and guidance for the better development of university library teaching in the future, provides better solutions for dealing with emergencies and critical teaching, provides teaching examples for exploring the deep integration of university library teaching and information technology, provides reference for better exploring the reform of university library teaching mode, plays a positive role in the good development of education, and has profound practical significance for understanding the profound influence of science and technology on teaching reform. Taking the teachers, students, and parents of library and information major in a university as the investigation objects, through oral research and interview, we can objectively and accurately understand the online teaching situation of the university library during the COVID-19 epidemic. Before the interview and investigation, determine the questions and make the interview records in time, so that the investigators can accurately capture the information, fully understand the facts, collect factual information according to the interview and investigation, and help the research work of the paper. This paper puts forward the construction of the online teaching acceptance model of university libraries under the epidemic situation, constructs the basic theoretical framework, establishes the basic evaluation indicators, takes the online teaching quality evaluation and the operability of the evaluation system as the constraint object, sets the index parameter set, determines the information of various online teaching resources at all levels, and conducts guidance and training with the three modules of preliminary preparation, online classroom and after-class review. The big data analysis based on the evaluation index system calculates the accurate teaching quality score or grade and realizes the online teaching acceptance evaluation of university libraries. The results of empirical analysis show that the model can realize the accurate evaluation of teaching quality, promote the deep integration of online teaching theory and practice in university libraries, and improve the acceptance level of online teaching quality.

## 2. Evaluation Index System of Online Teaching Acceptance of University Library under Epidemic Situation

### 2.1. Questionnaire Method and Online Teaching Quality Evaluation Index Parameter Model

15 experts and scholars from library science major of a university, and 5 external experts and scholars were selected to conduct a questionnaire survey. The 20 experts and scholars were selected as the research objects. Since the consent of all experts was obtained in advance, 20 questionnaires were distributed, and all valid questionnaires were collected, with a total of 20 questionnaires. The recovery rate was 100%. The reliability test of the questionnaires was conducted by the test-retest reliability analysis method. The purpose of the questionnaire survey is to understand the survey objects through the closed-ended and open-ended questions on the questionnaire. With the help of this tool, the researchers accurately and concretely measure the online teaching acceptance of the library, describe and analyze the quantity, and obtain the required survey data.

After completing the expert questionnaire, 10 experts were randomly selected from the respondents of the expert questionnaire at intervals of 10 days, and the same questionnaires were distributed again. The data collected from the two questionnaires were analyzed and sorted out. The results were as follows: experts unified the opinions of students, and students hoped that the library would provide information services for key majors and key courses, accounting for 36.97%; Tracking scientific research and providing information services, accounting for 19.70%; Regularly compile and print special reference materials, accounting for 25.15%; Providing users with proxy search, proxy connection, proxy copy, etc., accounting for 18.18%; The correlation coefficient R = 0.87 was obtained, which confirmed the reliability of the questionnaire data.

In this study, it is one of the most commonly used scientific research methods to screen and weight indicators. The questionnaire designed in advance was distributed to scholars and experts in library colleges, and each of them gave his own opinions and judgments on the same academic problem. In order to prevent the influence of other experts' suggestions, the opinions are expressed anonymously, and there is no connection between the experts. Finally, the suggestions of each expert are summarized. After repeated filling, the high convergence of expert suggestions is maintained in terms of results. In the process of this research, the deep integration of theory and practice has been realized. The theoretical route is as follows: based on the analysis of online teaching theory and practice at home and abroad, the theoretical basis and logical framework of this research are discussed from the key factors and motivations that affect the evaluation of teaching quality in university libraries. Systematic analysis, from the perspectives of pedagogy, evaluation, school library, and other disciplines, analyzes the conceptual connotation and theoretical support of online teaching quality evaluation in university libraries. The research roadmap is shown in Figure 1.

According to Figure 1, we can understand the current situation of the library, sort out the development of online teaching quality evaluation of university libraries through questionnaires and case studies, and understand the actual needs of teachers, students, and managers, thus laying a solid empirical foundation for the subject research. According to the results of theoretical research and empirical research, through logical analysis, this paper systematically analyzes the online teaching quality evaluation index system of university library courses and probes into its operability.

### 2.2. Integration of Online Teaching Acceptance Evaluation Parameters in University Libraries under the Epidemic Situation

In the evaluation indicators of layered teaching, there are mainly the following evaluation methods: the main body of evaluation is divided into others' evaluation and self-evaluation; The evaluation is divided into relative evaluation and absolute evaluation according to the evaluation reference standard; The time of evaluation is divided into pre learning, learning and post learning evaluation. There are various evaluation methods. When evaluating hierarchical teaching, we cannot use a single evaluation method, but use multiple methods to evaluate scientifically. The specific principles of evaluation are: the foothold of education is the evaluation and examination of students. In order to carry out the evaluation index model of layered teaching, we must innovate the evaluation mechanism of achievements. We should break the traditional quality evaluation concept of “one test paper for life” and establish an incentive mechanism for diversified evaluation. It combines the summative evaluation with the formative evaluation, and unifies the evaluation of students' academic achievements with the evaluation of learning attitudes and values. As a course, teaching includes students' theoretical lessons, practical lessons, and ordinary performances. Therefore, when evaluating a student's learning effect, we should not evaluate the student from one aspect of the student but should evaluate the student's learning effect from many aspects.

The basic theoretical framework of the online teaching evaluation system of university libraries under the epidemic situation is constructed, and the basic evaluation indexes are established. With the online teaching quality evaluation and the operability of the evaluation system as the constraint object, the index parameter set is combined and sorted with the horizontal distribution sequence of the acceptance estimation index samples. The mathematical description of the constrained optimization objective problem is as follows:

(1) $$\begin{array}{c} \mathrm{5628711.eq-inline.001} \end{array}$$

wherein *f*_*i*_(*x*) (*i* = 1, 2, ⋯, *n*) is the objective function of online teaching acceptance estimation of university libraries under the epidemic situation, *g*_*i*_(*x*) is the inequality constraint condition, and *h*_*j*_(*x*) is the correlation statistical constraint condition. This paper introduces the ambiguity detection technology of online teaching characteristics distribution in university libraries under the epidemic situation, and estimates the acceptance of online teaching in university libraries under the epidemic situation. In the process of this research, the deep integration of theory and practice has been realized. The theoretical route is as follows: based on the analysis of online teaching theory and practice at home and abroad, the theoretical basis and logical framework of this research are discussed from the key factors and motivations that affect the evaluation of teaching quality in university libraries [11, 12]. Systematic analysis, from the perspectives of pedagogy, evaluation, school library, and other disciplines, analyzes the conceptual connotation and theoretical support of online teaching quality evaluation in university libraries. The route of empirical research is: understanding the current situation of libraries, combing the development of online teaching quality evaluation of university libraries in China through questionnaires and case studies, and understanding the actual needs of teachers, students and administrators, thus laying a solid empirical foundation for the research. Finally, according to the results of theoretical research and empirical research, through logical analysis, this paper systematically analyzes the online teaching quality evaluation index system of university library courses in China, and probes into its operability [13–15].

**Definition 1 .**

The dominating set of online teaching acceptance estimation in university libraries under epidemic situation: the decision variable *x*^∗^ dominates *x* in online teaching acceptance estimation in university libraries under epidemic situation: all *x*, and there is at least one *f*_*i*_(*x*^∗^)<*f*_*j*_(*x*), where =1,2,…, n. At this time, the dominating set of autocorrelation fuzzy state of online teaching acceptance estimation in university libraries under epidemic situation satisfies local convergence.

**Definition 2 .**

Pareto optimal solution: for the discriminant statistic *X*^∗^ ∈ *S* of online teaching acceptance estimation of university libraries under epidemic situation, if and only if there is a boundary constraint solution *X* ∈ *S*, all inequalities are established, where *f*_*i*_(*X*^∗^) ≤ *f*_*i*_(*X*) D in the distribution range of online teaching acceptance of university libraries under epidemic situation, there is an *i*, This makes the characteristic distribution of online acceptance estimation of university library satisfy the strict inequality *f*_*i*_(*X*^∗^) < *f*_*i*_(*X*), and the statistics of online acceptance estimation of university library in epidemic background is a multi-objective optimization problem. By obtaining the Pareto optimal solution of the objective function of online acceptance estimation of university library in epidemic background, the convergence of the estimation model can be satisfied [16, 17].

## 3. Optimization of Online Acceptance Estimation Model of University Library under Epidemic Situation

### 3.1. Quantitative Analysis of Online Teaching Acceptance of University Libraries in the Context of Epidemic Situation

Establish a hierarchical analysis structure model based on the evaluation method, evaluation process and evaluation index system, determine the information of various online teaching resources at all levels, and give the constraint function of acceptance estimation [18–20]. Initialize the characteristic parameters of the acceptance estimation, modify the redundant vector set in the conclusion to obtain the optimal constraint index parameter *Pbest*, and determine the ambiguity function of the online teaching acceptance estimation of university libraries under the epidemic situation. The expression is

(2) $$\begin{array}{c} V_{ij}\left(g+1\right)=V_{ij}\left(g\right)+c_{1}r_{1ij}\left(g\right)\left[{Pbest}_{ij}\left(g\right)-x_{ij}\left(g\right)\right]+c_{2}r_{2ij}\left(g\right)\left[{Gbest}_{j}\left(g\right)-x_{ij}\left(g\right)\right], \end{array}$$

wherein *V*_*ij*_(*g*) is the joint estimation parameter of evaluation index and evaluation function, *c*_1_ is the fitness factor, *r*_1*ij*_(*g*) is the ambiguity coefficient, *Pbest*_*ij*_(*g*) is the fitness explanation parameter, *x*_*ij*_(*g*) is the statistical probability density function, and *Gbest*_*j*_(*g*) is the autocorrelation feature distribution set [21]. The learning model of online teaching acceptance estimation of university libraries under epidemic situation is set, and the number of nodes and vector elements *k* of online teaching acceptance distribution of university libraries under epidemic situation are obtained through fuzzy mathematical model [22, 23]. The autocorrelation feature distribution vector of online teaching acceptance estimation of university libraries under epidemic situation is:

(3) $$\begin{array}{c} x\left(t\right)={\left(x_{0}\left(t\right),x_{1}\left(t\right),\cdots ,x_{k-1}\left(t\right)\right)}^{T}, \end{array}$$

wherein *x*_0_(*t*), *x*_1_(*t*), ⋯, *x*_*k*−1_(*t*) is the subsequence of online teaching acceptance evaluation of university libraries. Combining with the association rule mining method, the formal distribution feature set of the association rule mining problem of online teaching acceptance evaluation of university libraries under epidemic situation is given [24, 25], and the weighted vector of online teaching acceptance evaluation of university libraries under epidemic situation is obtained as follows:

(4) $$\begin{array}{c} {Gbest}_{i}\left(g+1\right)=\arg_{{Pbest}_{ij}}^{\min}f\left({Pbest}_{ij}\left(g+1\right)\right), \end{array}$$

wherein *f*(*Pbest*_*ij*_(*g* + 1)) represents the load balancing scheduling parameter, and *g* is the association rule item of acceptance evaluation. This paper establishes the constraint parameter model of online teaching acceptance evaluation of university libraries under the epidemic situation.

### 3.2. Big Data Mining of Online Acceptance Estimation of University Libraries in the Context of Epidemic Situation

To determine the information of online teaching resources at all levels of online teaching in university libraries under the background of the epidemic situation, provide guidance and training in the three parts of early preparation, online classroom and after-school review, analyze the hierarchical structural characteristics of teaching quality, and integrate data standardization [26]. The correlation factors between *X*_*i*_ and *X*_*j*_ in the characteristic distribution of online teaching acceptance of university libraries under the epidemic situation are described as the similarity between the two characteristic quantities of teaching acceptance, expressed as follows:

(5) $$\begin{array}{c} l\left(X_{i},X_{j}\right)=\left\|X_{i}-X_{j}\right\|, \end{array}$$

wherein *X*_*i*_ and *X*_*j*_, respectively, represent the statistical time distribution sequence, and the above-mentioned distance similarity level represents the difference degree of online teaching acceptance estimation of university libraries under the epidemic situation. Through local convergence learning, the optimized weight subset {*W*_*O*_}_*i*=1_^*N*−*m*−*a*^ and the fuzzy parameter distribution subset of online teaching acceptance estimation of university libraries under the epidemic situation are obtained. Optimizing the distribution structure of online teaching quality in university libraries under the background of post-epidemic situation is expressed as follows:

(6) $$\begin{array}{c} {\left\{W_{O}\right\}}_{i=1}^{N-m-a}=\left\{{\left\{x_{O}^{i}\right\}}_{i=1}^{N-m-a}\right\}, \end{array}$$

wherein *x*_*O*_^*i*^ is the optimization characteristic quantity, and {*x*_*O*_^*i*^}_*i*=1_^*N*−*m*−*a*^ is the price system, which defines the evaluation range. If (*N_f_*/*N*) < *δ* the sample attribute set of the evaluation index of online teaching quality of university library under epidemic situation is recorded as *w*′*Φ*(*x*_*i*_) by using big data mining technology. Through collaborative optimization method, the online teaching acceptance of university library under epidemic situation is evaluated by using stochastic simulation and association rule decision method, and the online acceptance evaluation model of university library under epidemic situation is established by combining stochastic simulation dynamic detection and maximum matching analysis method.

(7) $$\begin{array}{c} GD=\frac{\sqrt{\sum_{i=1}^{n}{d_{i}}^{2}}}{n}, \end{array}$$

wherein *d*_*i*_ is the evaluation standard adopted by quality evaluators, and *n* is the dynamic distribution set of acceptance. When *GD* = 0, the convergence formula of online acceptance estimation of university libraries under the epidemic background is expressed as follows:

(8) $$\begin{array}{c} DM=\frac{d_{e}+d_{b}+\sum_{i=1}^{n-1}\left|d_{i}-\sum_{i-1}^{n-1}d_{i}/n-1\right|}{d_{e}+d_{b}+\left(n-1\right)\left(\sum_{i=1}^{n-1}d_{i}/n-1\right)}, \end{array}$$

wherein, *d*_*e*_ is the extreme point in the online teaching acceptance distribution set of university libraries under the epidemic situation, and *d*_*b*_ is the edge dynamic optimization function. To sum up, combined with random simulation dynamic detection and maximum matching degree analysis method, the online teaching acceptance of university libraries under the epidemic situation was evaluated.

## 4. Empirical Analysis

At present, there are many components involved in the course of university library, and the related research results are also extremely rich. Experts and scholars show different perspectives, showing different research needs, so they will have different conclusions and suggestions on this understanding. Some scholars believe that three key elements should be covered in university library courses: teaching objectives, teaching methods and teaching effects. However, the research on the basic elements needs to be closely related to the particularity of the library discipline at first, because the library discipline needs not only theoretical knowledge but also practical training. Therefore, researchers generally believe that besides curriculum objectives, curriculum contents and curriculum resources, sports theory and practice should also be demonstrated. In view of this, the basic elements of university library courses can be classified into the following categories: teacher quality, teaching process, curriculum resources and curriculum effectiveness. The quality of online teaching is bound to be influenced by these four basic elements. The first-level evaluation index system includes four dimensions: online teaching environment, professional background of school education, core team, and teachers, that is, the initial online teaching acceptance evaluation index framework includes four first-level indicators and 18 second-level indicators. See Table 1 for the first-level indicators of online teaching acceptance evaluation of university libraries under the epidemic situation. See Table 2 for the distribution of second-level indicators.

It can be seen from Table 1 that the first level indicators of online teaching acceptance evaluation of university libraries under the epidemic situation are divided into teacher quality, teaching process, course resources, and course effect.

It can be seen from Table 2 that in the secondary index classification, professional teaching ability, online teaching ability, professional background, and online teaching attitude play an important role. According to the setting of the above index parameters, the scatter diagrams of the first level indicators, second level indicators, and third level indicators of online acceptance evaluation of university libraries under the epidemic background are shown in Figures 2–4, respectively.

It can be seen from Figures 2–4 that the distribution of the three grade indicators is scattered in the overall range, and the distribution is relatively uniform. In order to realize the accurate selection of evaluation indexes and construct a scientific index evaluation system, this study uses Delphi method to investigate 20 experts and scholars inside and outside the school, and it is implemented by questionnaire. In terms of questionnaire distribution, it is mainly distributed on the spot, supplemented by mail. Through the preliminary statistical analysis of the questionnaire results, the evaluation index of online teaching quality is preliminarily drawn up. After the first round of expert questionnaire, the statistical results are analyzed, and the first, second, and third-level indicators, which are 4 items, 18 items, and 58 items, respectively, are selected with an average value of ≥4.0. Then, the second screening is conducted and combined with expert suggestions; it is more appropriate to change the first-level indicator “curriculum resources” to “teaching resources”. Among the four secondary indicators included in the course effect, such as student satisfaction, lifelong library awareness, ability training, and achievement award, there are unreasonable structures, which need to be changed to teaching goal achievement, student satisfaction, ability training, and participation achievement, and the cultivation of lifelong library awareness should be included in the achievement of teaching goal. Under the second-level indicator “online teaching ability”, three-level indicators such as “being able to choose an appropriate online teaching platform according to the teaching content”, “controlling reasonable exercise load”, and “having targeted teaching methods” are added, and under the second-level indicator “student satisfaction”, three-level indicators such as “looking forward to attending library classes” and “students' feedback information is better” are added. The third-level index “can accurately explain the technical essentials of movements” is changed to “can accurately explain and demonstrate the essentials of movements”, while the third-level index “motivation to participate in the experience” is changed to “actively participate in the experience teaching process”. The estimated analysis results of online teaching acceptance parameters of university libraries under the epidemic situation are shown in Table 3, the acceptance evaluation results of the three methods are shown in Figures 5–7, respectively.

It can be seen from table 3 that in the online teaching quality evaluation index system, which is based on university library courses, the first-class indexes and their weight ranking are teaching resources, course effect, teachers' quality, and teaching process. The main reason for this result is that the current online teaching mode has realized the gradual improvement of the teaching quality evaluation standard, and the focus is not only on teaching quality. It also includes the individualized development of students and emphasizes the objective evaluation of the process and results. In the process of specific activities, it cannot only fully display the main status of students but also implement the humanistic thought, pay attention to the development of students' personalities, and cast the concept of lifelong library in this process.

From Figures 5–7, it can be seen that compared with the results of the acceptance evaluation of principal component analysis and the acceptance evaluation of autocorrelation matching analysis, the acceptance of this method is higher because this method provides guidance and training in the three parts of preliminary preparation, online class and after-class review. Through the developmental characteristic analysis of acceptance estimation, To a certain extent, it is beneficial to improve the acceptance by analyzing the hierarchical structure characteristics of online teaching quality of University Libraries under the epidemic situation and integrating the data standardization.

To sum up, the method of this paper constructs the online teaching acceptance model of the university library, realizes the accurate evaluation of the teaching quality, promotes the deep integration between the online teaching theory and practice of the university library, and improves the acceptance level of the online teaching quality.

## 5. Discussion and Analysis

### 5.1. Continuously Improve the Remote Service Support Capability

The long-distance service guarantee ability is an important embodiment of the service ability of university library. Off campus remote access to various digital resources is the core demand of teachers and students. Only through preparation in advance, accurate assessment, timely disposal and all-round response can we ensure the solution of remote access needs. Although various university libraries can guarantee the acquisition demand of teachers and students' periodical literature through various ways, the protection of electronic teaching materials and auxiliary resources is still relatively backward. Many universities cannot effectively provide teaching materials and auxiliary books required by online courses. Therefore, the construction of electronic teaching materials and auxiliary libraries is an effective guarantee to ensure the acquisition demand of readers' resources.

### 5.2. Continuously Improve the Operation Ability of New Media

Compared with the traditional ways for readers to obtain library information (such as face-to-face consultation, web page publicity, e-mail notification, poster posting, etc.), the new media played a great role in the publicity of emergency services during the epidemic. At home, students can get all kinds of notices from the library through the library's wechat official account, wechat group, wechat applet, and microblog. Excellent wechat push can greatly facilitate readers to quickly obtain the information they need and accurately grasp the various services of the library. The librarian can also be on duty online to solve the reader's consultation problems in real time through wechat. At present, the wechat tweets of many university libraries need to be strengthened in terms of content. Not only should the themes be more diverse, and a certain type of wechat tweets can be pushed into a fixed brand, but also special personnel should be arranged to be responsible for the operation of new media, further strengthen the personnel team and technical ability, and form a stable and efficient operation and maintenance team.

### 5.3. Continuously Strengthen Cooperation with Other Units

“Unity, cooperation and coordination” is another feature of library services during the epidemic. In addition to cooperating with other departments in the school in terms of policy, technology, and application, the library also needs to cooperate with the database providers outside the school to obtain the dynamic resources in a timely manner and ensure the stable and orderly use of resources through technical means. Collaborative cooperation can increase the influence of libraries, expand the scope of services, and is conducive to the sharing of resources and collaborative development. In the future, major university libraries need to further develop ideas, fully mobilize the advantages and resources of other departments, and connect relevant resources and services through information service technology. Only in this way can they help each other overcome difficulties in emergency services and provide services that satisfy readers.

## 6. Conclusions

With the rapid development of China's economy, education is also developing rapidly. The teaching concept has been greatly changed, which has led to the subversive change of teaching activities. Teachers are no longer the dominant role, and students are more and more prominent in them. At the level of innovation and development of the teaching evaluation system, the proportion of student evaluation is getting higher and higher. This is consistent with quality education and can fully implement the humanistic teaching concept. This paper puts forward the construction of online teaching acceptance model of university library under the background of epidemic situation and draws the following conclusions through research:

- in the current indicator system, the online teaching mode, online teaching feedback, in school online teaching resources and out of school online teaching resources with the secondary indicator weight of more than 0.20
- compared with other methods, the method of constructing the online teaching acceptance model of university library in this paper has a higher acceptance under the background of epidemic situation
- the construction of online teaching acceptance model in university library is of great significance

## Figures and Tables

**Figure 1:** Technology roadmap.

**Figure 2:** Scatter diagram of primary index distribution.

**Figure 3:** Scatter diagram of secondary index distribution.

**Figure 4:** scatter diagram of tertiary index distribution.

**Figure 5:** Evaluation results of acceptance of this method.

**Figure 6:** Acceptance evaluation results of principal component analysis.

**Figure 7:** Acceptance evaluation results of autocorrelation matching analysis.

**Table 1:** First-level indicators of online teaching acceptance evaluation of university libraries under the background of epidemic situation.

Primary index	Serial number
Teachers' accomplishment	Q1
Teaching process	Q2
Curriculum resources	Q3
Course effect	Q4

**Table 2:** Secondary indicators of online teaching acceptance evaluation of university libraries under the epidemic situation.

Index	Serial number	Contribution level	Confidence level	Support degree
Professional teaching ability	QH11	0.534	0.616	0.233
Online teaching ability	QH12	0.687	0.415	0.488
Professional background	QH13	0.479	0.864	0.492
Online teaching attitude	QH14	0.362	0.962	0.328
Teachers' morality and style in online teaching	QH15	0.991	0.344	0.833
Online teaching research level	QH16	0.632	0.006	0.862
Online teaching content	QH17	0.665	0.002	0.842
Online teaching method	QH18	0.961	0.539	0.839
Online teaching mode	QH19	0.135	0.712	0.534
Online teaching management	QH20	0.841	0.266	0.510
Online teaching feedback on campus	QH21	0.800	0.669	0.460
Online teaching resources off campus	QH22	0.201	0.846	0.624
Online teaching sprang from construction.	QH23	0.988	0.322	0.202
Online resource student satisfaction	QH24	0.316	0.940	0.105
Cultivate lifelong learning awareness and ability	QH25	0.543	0.476	0.635
Achievement award	QH26	0.024	0.504	0.222
Examination	QH27	0.980	0.071	0.822

**Table 3:** Estimation and analysis of online teaching acceptance parameters of university libraries under the background of epidemic situation.

Test object	Library practice teaching investment	Practical classroom teaching effect in library	Student satisfaction level	Regression analysis value
QH11	0.176	0.282	0.940	0.176
QH12	0.997	0.762	0.678	0.997
QH13	0.015	0.359	0.227	0.015
QH14	0.261	0.346	0.888	0.261
QH15	0.418	0.454	0.081	0.418
QH16	0.251	0.120	0.991	0.251
QH17	0.637	0.804	0.192	0.637
QH18	0.408	0.631	0.657	0.408
QH19	0.543	0.677	0.595	0.543
QH20	0.876	0.250	0.544	0.876
QH21	0.721	0.309	0.494	0.721

## Data Availability

The raw data supporting the conclusions of this article will be made available by the authors, without undue reservation.
